# Glycoprotein non-metastatic melanoma B interacts with epidermal growth factor receptor to regulate neural stem cell survival and differentiation

**DOI:** 10.1515/med-2023-0639

**Published:** 2023-02-14

**Authors:** Hua Yang, Gang Jin, Shihong Chen, Jing Luo, Wei Xu

**Affiliations:** Department of Rehabilitation, Taizhou Central Hospital (Taizhou University Hospital), Taizhou, China; Orthopedics Department, Taizhou Hospital of Zhejiang Province Affiliated to Wenzhou Medical University, Linhai City, Taizhou, Zhejiang Province, 317000, China

**Keywords:** glycoprotein non-metastatic melanoma B, epidermal growth factor receptor, spinal cord injury, functional recovery, cell differentiation

## Abstract

The functional recovery following spinal cord injury (SCI) remains a challenge clinically. Among the proteins interacted with the *glycoprotein non-metastatic melanoma B (GPNMB)*, *epidermal growth factor receptor (EGFR)* during activation is able to promote the proliferation of neural stem cells (NSCs) in the spinal cord. We investigated the roles of *GPNMB* and *EGFR* in regulating the survival and differentiation of the NSCs. By overexpression and short-hairpin RNA-mediated knockdown of *GPNMB* in the NSCs, *GPNMB* promoted cell viability and differentiation by increasing the expressions of βIII tubulin and CNPase (2′,3′-cyclic nucleotide 3-phosphodiesterase). Using co-immunoprecipitation, we found that *EGFR* interacted with *GPNMB*. Furthermore, *EGFR* had a similar effect as *GPNMB* on promoting cell viability and differentiation. Overexpression of *EGFR* reversed the decrease in viability and differentiation caused by the knockdown of *GPNMB*, and *vice versa*. Last but not least, we tested the effect of GPNMB and EGFR on several intracellular pathways and found that *GPNMB/EGFR* modulated the phosphorylated (p)-c-Jun N-terminal kinase (JNK)1/2/JNK1/2 ratio and the p-nuclear factor κB (NF-κB p65)/NF-κB p65 ratio. In sum, our findings demonstrate the interaction between *GPNMB* and *EGFR* that regulates cell bioprocesses, with the hope to provide a new strategy of SCI therapy.

## 1 Introduction

Spinal cord injury (SCI) has been emerged as a serious and irreversible disease in the central nervous system (CNS) [1], bringing about permanent or temporary loss of function in the motor or sensory capability and leading to destructive neurological and functional deficiency inclusive of paraplegia or quadriplegia [2]. Due to the lack of regeneration capacity, the recovery of the body function as impaired by SCI remains a significant challenge clinically [3]. In this case, the efforts devoted into exploring the functions of endogenous spinal cord neural stem cells (NSCs) shed a light on the treatment of SCI [4,5].

NSCs, primarily indwelling in the CNS including the spinal cord and the brain, are competent to self-renew for the maintenance of the stem cell bank size and to differentiate into neurons for the repairmen of the tissues [4,6], which is likely to be distinguished in the functional recovery of SCI. Given the inclination of NSCs to differentiate into microenvironment-dependent glia lineages, many researchers have committed to facilitating the differentiation into functional neurons from the spinal cord neural progenitor cells (NPCs) [7,8].

The differentiation inducement attempts involve the regulation of the proteins in the spinal cord to trigger the endogenous repair [9]. We started our study by analyzing transcriptome changes via the aberrant gene expressions either in the young or aged patients perplexed by SCI based on the data set GSE93561 and captured 90 genes expressing aberrantly after crossover analysis. Glycoprotein non-metastatic melanoma B (GPNMB) has aroused our interest by dint of its multiple functions, encompassing tissue repairment facilitation, kinase signaling stimulation, cell–cell adhesion and migration acceleration, tumorigenesis promotion, modulation of the cell growth and differentiation, etc. [10]. *GPNMB* is a type I transmembrane glycoprotein [11], whose expression level is found upregulated in SCI according to the analyses of the above-mentioned data set. Apart from that, *GPNMB* also exhibits dysregulated expression in the spinal cord transcriptome after peripheral nerve injury [12] and in a high-fat diet-fed male rat model of thoracic spinal contusion [13]. However, the regulatory mechanism of *GPNMB* in SCI remains uncharacterized.

To figure out the regulatory mechanism of *GPNMB* in SCI, we adopted bioinformatics analysis to predict the proteins interacting with *GPNMB*. Notably, *epidermal growth factor receptor* (*EGFR*), a transmembrane glycoprotein of ErbB family, was finalized, given that the activation of *EGFR* contributed to the proliferation of NSCs in SCI [14]. *EGFR* signaling cascade features in the proliferation, division, differentiation, and survival of the cells [15]. It has been elucidated that *EGFR* can regulate a variety of downstream pathways, including Janus kinase/signal transducer and activator of transcription, extracellular signal-regulated kinase/mitogen-activated protein kinase, phosphatidylinositol 3-kinase (PI3K)/Akt, and Notch pathways, and promote the NSC proliferation [16,17,18]. *EGF* (*epidermal growth factor*), a ligand of *EGFR*, activates *EGFR* and enhances the proliferation of local NSCs, playing an active role in SCI [19]. In line with the above findings, we are dedicating to validating whether *GPNMB* interacts with *EGFR* to regulate cell survival and differentiation in SCI, so as to provide a novel insight for the further prognosis for SCI patients.

## 2 Methods

### 2.1 Ethics statement

All the research studies related to animal use were complied with the relevant national regulations and institutional policies for the care and use of animals. This study was conducted on the premise of authorization from the Ethic Committee of Experimental Animals of Taizhou Central Hospital (Taizhou University Hospital) with approval number SJWK202001010. Every effort was exploited to minimize the pain and discomfort to the animals.

### 2.2 Bioinformatics analysis

SCI microarray data were downloaded from the gene expression omnibus database (http://www.ncbi.nlm.nih.gov/geo/) using the accession number, GSE93561 (https://www.ncbi.nlm.nih.gov/geo/query/acc.cgi?acc=GSE93561) [20]. Search tool, the Retrieval of Interacting Genes Database (STRING) (https://www.string-db.org/), was adopted to comprehensively analyze the data for protein–protein interaction (PPI) network [21].

### 2.3 Neurosphere culture

Before the operation, the C57BL/6 mice neonates (<12 h after birth) from five pregnant C57BL/6 mice (C57BL/6JNifdc; Charles River Laboratories, Wilmington, MA, USA) in this study were anesthetized with ketamine (80 mg/kg; K-002; Sigma-Aldrich) and intraperitoneally injected with xylazine (10 mg/kg, X1126; Sigma-Aldrich). Next, T10 spinal cord was exposed after the removal of the vertebral lamina and then completely cut by the scissors. NPCs were obtained as previously described [3]. The cut-off spinal cords were then dissociated by TrypLE Express (12604013; Gibco, USA) at 37°C for 25 min. Subsequently, the single-cell suspension of the NPCs was placed in Dulbecco’s modified Eagle’s medium (DMEM)/F-12 (31331093; Gibco) supplemented with 1% penicillin–streptomycin antibiotics (15240096; Gibco), 2% B27 (A3582801; Gibco), 20 ng/mL EGF (AF-100-15; PeproTech, New Jersey, USA), and 20 ng/mL fibroblast growth factor-basic (bFGF; AF-100-18B; PeproTech). Afterward, the neurospheres were digested by Trypsin (R001100; Gibco) digestion buffer in the subsequent experiments and cultured in DMEM with high glucose (DMEM-H; 11995040; Gibco) supplemented with 10% fetal bovine serum (FBS; 12664025; Gibco).

### 2.4 NPC differentiation

NPC differentiation inducement was implemented as previously described [22]. Briefly, cells were digested and resuspended into single-cell suspension, followed by the seeding in culture dishes coated with poly-l-lysine (P4707; Sigma-Aldrich). Thereafter, cells were cultured in DMEM/F-12 medium supplemented with 2% B27 and 1% FBS to induce differentiation. The culture medium was replaced every 2 days. NPCs cultured in DMEM/F-12 medium without any treatment served as the control group.

### 2.5 Cell transfection

Cells were initially transfected with overexpressed plasmid of *GPNMB*, short-hairpin RNA (shRNA) targeting *GPNMB* (shGPNMB) and their negative controls (shNC) [21], and subsequently continued for transfection with EGFR overexpression plasmid and shRNA targeting *EGFR* (shEGFR). Overexpressed plasmids for *GPNMB* or *EGFR* were constructed by inserting the whole sequences of *GPNMB* or *EGFR* into pcDNA 3.1 empty vector (V79020; Thermo Fisher Scientific, Waltham, MA, USA). Empty vector was used as NC (negative control). ShNC, shGPNMB (5′-TGAGGGAGCACAATCAATTAA-3′), shGPNMB (shRNA#2; 5′-GTGTACATATTCTACTCATTA-3′), shGPNMB (shRNA#3; 5′-GGAGCTTTGTCTACGTCTTTC-3′), shEGFR (5′-GAATAGGTATTGGTGAATTTA-3′), shEGFR (shRNA#2; 5′-GCATAGGCATTGGTGAATTTA-3′), and shEGFR (shRNA#3; 5′-CCAAGCCAAATGGCATATTTA-3′) were all synthesized by GenePharma (Shanghai, China). Before transfection, cells were cultured in six-well plates (CLS3335, Corning, NY, USA) till 90% confluence was reached. Prior to transfection, the culture medium was removed and cells were washed with phosphate-buffered saline (PBS) (806552; Sigma-Aldrich) and then transfected with commercially available GenePharma substances via Lipofectamine 2000 transfection reagent (11668027; Invitrogen, CA, USA). Briefly, 50 nanogram/mol (nM) shGPNMB, shEGFR or NC and 10 μL Lipofectamine reagent were diluted in 250 μL serum-free DMEM, and then cultured in the Opti-MEM™ medium (11058021; Thermo Fisher Scientific) at room temperature for 5 min. After the addition of DNA–lipid complex, cells were incubated at 37°C for 24 h before analysis.

### 2.6 Western blot assay

Protein expression levels of βIII tubulin, 2′,3′-cyclic nucleotide 3′-phosphodiesterase (CNPase), GPNMB, EGFR, c‑Jun NH2‑terminal kinase (JNK)1/2, phosphorylated (p)-JNK1/2 (p-JNK1/2), and nuclear factor κB (NF-κB) p65 were measured by Western blot assay, with glyceraldehyde-3-phosphate dehydrogenase (GAPDH) as the internal reference. Simply put, cells were harvested and extracted by 300 μL RIPA lysis buffer (20-188; Sigma-Aldrich) containing protease and phosphatase inhibitor (P1045; Beyotime, Shanghai, China), followed by the centrifugation for collection of supernatant. Thereafter, concentrations of proteins in the supernatant were measured by a bicinchoninic acid kit (P0011; Beyotime) based on manufacturer’s directions. Subsequently, the proteins with equal weight of 30 µg were electrophoresed on 10% sodium dodecyl sulfate polyacrylamide gel electrophoresis (SDS-PAGE) and then transferred onto the polyvinylidene fluoride (PVDF) membrane (FFP28; Beyotime). The membrane was blocked with 5% skimmed milk at room temperature for 1 h and then incubated with the primary antibodies at 4℃ overnight. Herein, the varied primary antibodies included anti-βIII tubulin (rabbit, 1:1,000, 50 kDa, ab18207; Abcam, Cambridge, UK), anti-CNPase (rabbit, 1:1,000, 48 kDa, ab250658; Abcam), anti-GPNMB (rabbit, 1:5,000, 120 kDa, ab188222; Abcam), anti-EGFR (rabbit, 1:2,000, 175 kDa, ab52894; Abcam), anti-JNK1/2 (mouse, 1:500, 54 kDa, sc-137019; Santa Cruz, Texas, USA), anti-p-JNK1/2 (rabbit, 1:1,000, 46–54 kDa, ab124956; Abcam), anti-NF-κB p65 (rabbit, 1:1,000, 65 kDa, ab32536; Abcam), anti-p-NF-κB p65 (rabbit, 1:1,000, 65 kDa, ab239882; Abcam), and anti-GAPDH (mouse, 1:500, 36 kDa, ab9484; Abcam). Afterward, the membranes were thereupon incubated with horseradish peroxidase-conjugated secondary antibodies goat anti-rabbit IgG (1:3,000, ab205718; Abcam) and goat anti-mouse IgG (1:3,000, ab6789; Abcam) at room temperature for 2 h. Protein signals were tested and collected via the enhanced chemiluminescence Kit (P0018S; Beyotime) and quantified through ImageJ software (ImageJ 1.8.0; Bethesda, MD, USA).

### 2.7 Quantitative reverse-transcription polymerase chain reaction (qRT-PCR)

Relative *GPNMB* and *EGFR* mRNA expression levels were measured by qRT-PCR. Briefly, total RNAs were extracted via TRIzol reagent (15596026; Invitrogen), whose quantities and purities were determined by a spectrophotometer (ND-LITE-PR; Thermo Fisher Scientific) and transcribed reversely by an RNA transcriptase kit (K1621; Thermo Fisher Scientific) based on the manufacturer’s instructions. qRT-PCR experiment was carried out with the SYBR PremixEx Taq II Kit (RR820L; TaKaRa, Japan) in LightCycler 480-II System (Roche Diagnostics, Penzberg, Germany). The qRT-PCR amplification conditions were listed as follows: 95℃ for 5 min; 40 cycles at 95℃ for 5 s, 60℃ for 20 s, and 72°C for 40 s. Primer sequences for *GPNMB* were 5′-ACTTGGGCCTCAACTCATGG-3′ (Forward) and 5′-GCAGGTGGGGTCAGAAATGA-3′ (Reverse). Primer sequences for *EGFR* were 5′-TCTCCAAAATGGCCCGAGAC-3′ (Forward) and 5′-CAGGATTCTGCACAGAGCCA-3′ (Reverse). Primer sequences for *GAPDH* were 5′-TTCACCACCATGGAGAAGGC-3′ (Forward) and 5′-GATGGCATGGACTGTGGTCA-3′ (Reverse). For results calculations, 2^−ΔΔCt^ method was adopted [23] with *GAPDH* as the internal reference.

### 2.8 Cell counting kit-8 (CCK-8) assay

Cell viability was measured by CCK-8 assay kit (C0037; Beyotime) following the manufacturer’s instructions. Cells were first seeded into 96-well plates (CLS3922; Corning) at a density of 4 × 10^4^ cells per well for 24, 48, and 72 h. Subsequently, 10 µL of CCK-8 solution was added into every well for further 2-h incubation. Afterward, the optical density (OD) was assessed at a wavelength of 450 nm via a microplate reader (Varioskan LUX; Thermo Fisher).

### 2.9 Immunofluorescence

Cells were immobilized with 4% precooling paraformaldehyde (P1110; Solarbio, Beijing, China) for 30 min and permeabilized with 0.3% Triton X-100 (T8200; Solarbio) at room temperature for 10 min. After being blocked in 1% bovine serum albumin (BSA; A8020; Solarbio) for 30 min, cells were incubated with primary antibodies including anti-βIII tubulin (1 μg/mL) and anti-CNPase (5 µg/mL) at 4℃ overnight. Post three times of washing in PBS (806552; Sigma-Aldrich), the primary antibodies were identified with Alexa Fluor 594 goat-anti rabbit antibodies (B40925; Invitrogen) for 60-min incubation at room temperature. Subsequently, the nuclei were counter-stained with DAPI (C1002; Beyotime) at 37℃ for 10 min. Ultimately, the slides were mounted and observed under a fluorescence microscope (Leica, TCS SP5II, Germany).

### 2.10 Co-immunoprecipitation (Co-IP) assay

Co-IP assay was implemented utilizing the Pierce Co-IP Kit (26149; Thermo Fisher Scientific) following the manufacturer’s instructions. In a nutshell, the harvested cells were homogenized by ice-cold non-denaturing lysis buffer (25 mM Tris, 150 mM NaCl, 1 mM EDTA [ethylenediamine tetra acetic acid], 1% Nonidet P-40 [NP-40] and 5% glycerol; pH 7.4) with the addition of 2× complete protease inhibitor cocktails (11206893001; Roche, Mannheim, Germany) and then centrifuged for 20 min. The supernatant was collected and the protein concentration was quantified. A 50 μL aliquot of cell lysate was saved as the input, and the resulting supernatant was pre-cleaned for 1-h incubation with Pierce Control Agarose Resin at 4℃. Subsequently, the antibody against GPNMB (1:30) or EGFR (1:20) was incubated with AminoLink Plus coupling Resin for 2 h and washed three times with the Coupling Buffer (10 mM sodium phosphate, 150 mM NaCl; pH 7.2). Meanwhile, the antibody against IgG was set as the NC. The pre-cleaned lysates (1 mg of proteins) were incubated with antibody-coated Resin at 4℃ for 2 h. After being washed three times with the lysis buffer, the precipitates were separated on SDS-PAGE for Western blot analysis and probed with anti-GPNMB or anti-EGFR antibody, respectively.

### 2.11 Statistical analysis

All values were presented as mean ± standard deviation (SD). Independent samples *t* test was applied for the analysis between two variables. One-way analysis of variance was adopted to analyze one categorical independent variable in multiple groups, followed by Bonferroni post hoc analysis. GraphPad Prism 8 software (GraphPad, CA, USA) was utilized for data analysis. For measurements, *P* < 0.05 was perceived as statistical significance.

## 3 Results

### 3.1 *GPNMB* promoted neuronal viability and differentiation while shGPNMB performed differently

Post bone marrow NSC extraction and differentiation inducement, we utilized Western blot assay to detect the differentiation degree of the cells. Upregulated protein expression of the neural differentiation marker, βIII tubulin, indicated the successful differentiation of NSCs into neurons (Figure 1a, *P* < 0.001). Then, we measured *GPNMB* expression changes after cell differentiation via qRT-PCR and Western blot assay. Results from both assays demonstrated that *GPNMB* expression level was upregulated in the differentiated cells relative to that in control cells (Figure 1b and c, *P* < 0.001). Next, we transfected the cells with the overexpressed or silenced *GPNMB* plasmid to figure out the impact of *GPNMB* upon cell viability and neural differentiations. shGPNMB was used for further experiment due to its more efficiency of *GPNMB* knock down (Figure A1a, *P* < 0.01). Moreover, qRT-PCR and Western blot assays demonstrated that overexpressed *GPNMB* promoted while shGPNMB reduced *GPNMB* expression, indicating the success of transfection (Figure 1d–e, *P* < 0.001). Besides, CCK-8 assay manifested that *GPNMB* overexpression boosted cell viability; yet, shGPNMB restrained cell viability in the endured test time (Figure 1f, *P* < 0.05). Finally, neural differentiation was assessed by the immunolabeling profiles of the neuronal marker βIII tubulin and oligodendrocyte marker CNPase [24], followed by the measurement of Western blot assay, the results of which displayed that overexpressed *GPNMB* upregulated βIII tubulin and CNPase expression levels (Figure 1g–h, *P* < 0.05), whilst shGPNMB downregulated the expressions of the neural differentiation markers (Figure 1g–h, *P* < 0.001).

**Figure 1:** *GPNMB* promoted cell viability and neuronal differentiation while shGPNMB performed differently. (a) Relative βIII tubulin expression was measured by qRT-PCR and Western blot assay. Upregulation of βIII tubulin expression suggested the successful differentiation of the neural stem cells into neurons. (b and c) Relative *GPNMB* expression was measured by qRT-PCR and Western blot assay. (d and e) Transfection efficiency was validated by qRT-PCR and Western blot assay. (f) Cell viability was measured via CCK-8. *GPNMB* promoted while shGPNMB inhibited cell viability. (g) Immunofluorescence assay was adopted to assess the status of neuronal differentiation (magnification 200×, scale bar 100 µm). Red part referred to the targeted proteins, and blue meant the nuclei as stained by DAPI. (h) Relative neural differentiation markers’ (βIII tubulin and CNPase) expressions were measured by Western blot assay. *GAPDH* was set as the internal reference. ^**^ *P* < 0.01 or ^***^ *P* < 0.001 vs Control; ^+^ *P* < 0.05 or ^+++^ *P* < 0.001 vs NC; ^##^ *P* < 0.01, ^###^ *P* < 0.001 vs shNC. All results represent means ± SD of triplicate determinations. qRT-PCR: quantitative reverse-transcription polymerase chain reaction; *GPNMB*: *glycoprotein non-metastatic melanoma B*; shNC: short-hairpin-negative control; CCK-8: cell counting kit-8; CNPase: 2′,3′-cyclic nucleotide 3′ phosphodiesterase.

### 3.2 *EGFR* interacted with *GPNMB* and its expression level was upregulated in the differentiated cells

To figure out the regulatory mechanism of *GPNMB*, we adopted STRING to analyze the proteins interacting with GPNMB (Figure 2a). Ultimately, EGFR was selected as the candidate on the basis of literature study. To validate the interaction between GPNMB and EGFR, we performed Co-IP assay with identification that GPNMB coprecipitated with EGFR (Figure 2b and c). Then, we conducted qRT-PCR and Western blot assay again to measure the expression level of *EGFR* and discovered that *EGFR* was upregulated in the differentiated cells relative to that in control cells (Figure 2d–e, *P* < 0.001).

**Figure 2:** *EGFR* interacted with *GPNMB* and its expression level was downregulated after cell differentiation. (a) STRING (https://www.string-db.org/) was adopted to comprehensively analyze the data for PPI network. *GPNMB* interacted with *EGFR*. (b and c) A Co-IP assay was performed to identify if *GPNMB* coprecipitated with *EGFR*. (d and e) Relative *EGFR* expression was measured by qRT-PCR and Western blot assay. *GAPDH* was set as the internal reference. ^**^ *P* < 0.01 ^***^ *P* < 0.001 vs control. All results represent means ± SD of triplicate determinations. STRING: Retrieval of Interacting Genes Database; PPI: protein–protein interaction; *EGFR*: e*pidermal growth factor receptor*; Co-IP: co-immunoprecipitation.

### 3.3 *EGFR* boosted cell viability and partly reversed the effect of shGPNMB

Subsequently, we further explored the mechanism with the participation of aberrant *EGFR* expression through transfection. ShEGFR was used for next experiment because of its more efficiency of *EGFR* knock down (Figure A1b, *P* < 0.001). As supported by the measurements from qRT-PCR and Western blot assays, overexpressed *EGFR* upregulated *EGFR* expression, whereas shEGFR downregulated *EGFR* expression, which indicated the success of transfection (Figure 3a and b, *P* < 0.001). Then, we implemented CCK-8 assay to reveal the effect of *EGFR* on cell viability, finding that shEGFR suppressed cell viability; yet, *GPNMB* boosted cell viability and could partly reverse the inhibiting effect of shEGFR (Figure 3c, *P* < 0.05). Besides, shGPNMB restrained cell viability, while EGFR stimulated cell viability and partly counteracted the suppressive effect of shGPNMB (Figure 3d, *P* < 0.05).

**Figure 3:** *EGFR* facilitated cell viability and partly reversed the effect of shGPNMB. (a and b) Transfection efficiency was verified by qRT-PCR and Western blot assay. Overexpressed *EGFR* promoted *EGFR* expression but shEGFR reduced *EGFR* expression. (c and d) Cell viability was measured through CCK-8. GAPDH was used as the internal reference. ^***^ *P* < 0.001 vs NC; ^+++^ *P* < 0.001 vs shNC; ^^^ *P* < 0.05，^^^^^ *P* < 0.001 vs NC + shNC; ^##^ *P* < 0.01 vs GPNMB + shNC; ^&&&^ *P* < 0.001 vs NC + shEGFR; ^ε^ *P* < 0.05, ^εε^ *P* < 0.01, ^εεε^ *P* < 0.001 vs shNC + NC; ^ΩΩΩ^ *P* < 0.001 vs shGPNMB + NC; ^Δ^ *P* < 0.05, ^ΔΔ^ *P* < 0.01 vs shNC + EGFR. All results represent means ± SD of triplicate determinations. shEGFR: short-hairpin RNA-targeting *EGFR*.

### 3.4 *EGFR* facilitated p-JNK1/2/JNK1/2 ratio and NF-κB p65 expression and partly counteracted the inhibitory effects of shGPNMB on the JNK/NF-κB signaling pathway while shEGFR displayed oppositely

Then, we adopted the immunofluorescence assay to explore the status of neuronal differentiation after the second-phase transfection, followed by Western blot assay. The results uncovered that overexpressed *GPNMB* increased βIII tubulin and CNPase protein expressions, while shEGFR decreased βIII tubulin and CNPase expressions and could partly neutralize the promotive effects of *GPNMB* on the expressions of these two proteins (Figure 4a, *P* < 0.001). Moreover, shGPNMB lessened βIII tubulin and CNPase protein expressions, whereas *EGFR* enhanced βIII tubulin and CNPase expressions and partly offset the restraining function of shGPNMB in the above aspects (Figure 4b, *P* < 0.001). Finally, we validated our conjecture through detecting JNK/NF-κB signaling pathway-related indicators via Western blot assay. *GPNMB* boosted the p-JNK1/2/JNK1/2 ratio and the p-NF-κB p65/NF-κB p65 ratio, but shEGFR worked inversely and partly reversed the enhancing effects of *GPNMB* on JNK/NF-κB signaling pathway-related markers (Figure 4c, *P* < 0.05). On the contrary, shGPNMB reduced the p-JNK1/2/JNK1/2 ratio and the p-NF-κB p65/NF-κB p65 ratio; yet, *EGFR* facilitated these ratios and partly counteracted the inhibitory effect of shGPNMB on the JNK/NF-κB signaling pathway-associated markers (Figure 4d, *P* < 0.001).

**Figure 4:** *EGFR* up-regulated p-JNK1/2/JNK1/2 ratio and NF-κB p65 expression and partly offset the suppressive effect of shGPNMB on the JNK/NF-κB signaling pathway while shEGFR worked inversely. (a and b) Relative βIII tubulin and CNPase expressions were measured by Western blot assay. (c and d) Expressions of JNK/NF-κB signaling pathway-related indicators were measured by Western blot assay. *GAPDH* was employed as the internal reference. ^^^ *P* < 0.05 or ^^^^^ *P* < 0.001 vs NC + shNC; ^###^ *P* < 0.001 vs GPNMB + shNC; ^&&^ *P* < 0.01, ^&&&^ *P* < 0.001 vs NC + shEGFR; ^ε^ *P* < 0.05 or ^εεε^ *P* < 0.001 vs shNC + NC; ^Ω^ *P* < 0.05 or ^ΩΩΩ^ *P* < 0.001 vs shGPNMB + NC; ^ΔΔΔ^ *P* < 0.001 vs shNC + EGFR. All results represent means ± SD of triplicate determinations. JNK 1/2: c‑Jun NH2‑terminal kinase 1/2; p-JNK 1/2: phosphorylated JNK1/2; NF-κB p65: nuclear factor κB p65.

## 4 Discussion

In the present study, we found that *GPNMB* and *EGFR* formed PPIs and both proteins were downregulated in differentiated neuronal cells. In addition, *GPNMB* and *EGFR* have at least partial complementary functions, with one protein overexpression reversing the effects of the other protein silencing, including cell viability, differentiation, and JNK/NF-κB signaling activation.

GPNMB has aroused overriding interest from researchers by virtue of its aberrant expression in cancers and the correlation with multiple biological processes composing of tissues’ regeneration and cell differentiation [25]. As put forward by Spann et al., *GPNMB* is a promising objective for chronic SCI treatment, whose expression is upregulated in SCI [13]. Weng et al. further validated the upregulation of *GPNMB* in the spinal cord after sciatic nerve injury and its participation in the cellular events of growth and development [12]. Both of these findings verify the correlation of *GPNMB* with SCI, but the underlying mechanism remains elusive.

On the basis of a previous research, we further conducted our study on the perspective of functional recovery of SCI, which was impacted by the neuron loss in most occasions [3]. Generally, the main obstacle for SCI treatment would be the effective usage of the stimulated endogenous NPCs. A previous study stated *GPNMB* as a novel neuroprotective factor in cerebral ischemia–reperfusion injury [26]. Also, a recent study demonstrated that *GPNMB* could be a novel strategy for peripheral nerve regeneration after transection by promoting the proliferation of Schwann cells as well as expression and secretion of neurotrophic factors and neural adhesion molecules *in vitro* [27]. In our study, we uncovered that overexpression of *GPNMB* was beneficial to cell viability and neuronal differentiations as supported by the expression changes of the neural differentiation-associated markers (βIII tubulin and CNPase) *in vitro* which might avail the restricted recovery after SCI. We took over the studies against *GPNMB* from Spann et al. and Weng et al. and ulteriorly proved the possible role of *GPNMB* in SCI from the perspective of probing into the underlying regulation of cell differentiation rather than lingering on the surface.

As for the detailed mechanism, the interaction between *GPNMB* and *EGFR* in SCI, on the basis of a research reported by Han et al. who had already demonstrated *GPNMB* as an activator in cell migration, and its upregulation might be related to the oncogenic property of *EGFR* in lung cancer [28]. Despite the different study field and research direction, we substantiated the synergistic effect between *GPNMB* and *EGFR* in the non-cancer field and raised that the interaction between the two functioned in the biological processes and cell differentiation in NSCs. Liu et al. conducted a study on the individual role of *RGFR* in SCI and validated the promotive role of *EGFR* in NSC activation after SCI [14]. Similar to Liu et al., we also highlighted the significance of *EGFR* in NSC activation for functional recovery after SCI, although two of us focused on a different signaling pathway.

Fang et al. had confirmed the participation of JNK/NF-κB pathway in SCI through the inhibitory regulation of miR-132-3p on attenuating the injury [29]. It has been evidenced that NF-κB signaling pathway functions prominently in immune response and neuroinflammation; with a great detail, the neuroinflammation could be triggered by the NF-κB signaling pathway after SCI [30]. In addition, inactivation of this pathway can ameliorate the SCI via modulating the inflammatory reaction [31,32]. As for the JNK pathway, its significance has been validated in the contribution to the neuronal apoptosis after neuron injury [33,34]. In our study, we further confirmed the involvement of JNK/NF-κB signaling pathway in SCI and uncovered that GPNMB interacted with EGFR to modulate JNK phosphorylation and NF-κB p65 phosphorylation, thereby making an impact upon neuronal differentiation. This finding is a further extension of Fang et al. in SCI treatment and provides a novel cue in the regulatory mechanism of stimulating endogenous NPCs for SCI therapy. Typically, PI3K/protein kinase B (Akt) and RAS/RAF pathways are the main downstream pathways that EGFR regulates survival and differentiation. These two pathways are not detected in this study, which is the shortcoming of this study. Moreover, whether *GPNMB* regulates *EGFR* protein abundance and PI3K/Akt and whether RAS/RAF pathway affects the survival and differentiation of NSCs need further investigation. At present, the study of *GPNMB* is still in its infancy and the role of *GPNMB* in the multiple tumors or non-tumor cases requires to be further elucidated. Further studies toward *GPNMB* in SCI are welcomed and recommended to validate the performances and properties in the actual practice. Besides, the interaction between *GPNMB* and *EGFR* or other proteins is worth pursuing due to the extensive scope captured from the bioinformatics analysis. Furthermore, ulterior studies are expected to exploit the actual value of this interaction as therapeutic entity to induce NPCs in terms of feasibility and practicability.

In conclusion, we prove that the interaction between *GPNMB* and *EGFR* regulates neuronal survival and differentiation through the modulation of JNK/NF-κB signaling pathway.

## Figures and Tables

**Figure A1:** The efficiency of knock down for GPNMB and EGFR. (a) The knock down efficiency of shGPNMB, shGPNMB (shRNA#2) and shGPNMB (shRNA#3) for GPNMB. (b) The knock down efficiency of shEGFR, shEGFR (shRNA#2) and shEGFR (shRNA#3) for EGFR. GAPDH was set as the internal reference. ^++^*P* < 0.01 or ^+++^*P* < 0.001 vs. shNC. All results represent means of ±standard deviation (SD) of triplicate determinations. (qRT-PCR: quantitative reverse-transcription polymerase chain reaction; GPNMB: glycoprotein non-metastatic melanoma B; EGFR: epidermal growth factor receptor; shNC: short hairpin negative control).
